RETRACTED

# Percutaneous Aspiration Thrombectomy for Arterial Thromboembolism during Infrainguinal Endovascular Recanalization

**DOI:** 10.1371/journal.pone.0140494

**Published:** 2015-10-20

**Authors:** Li-Ming Wei, Yue-Qi Zhu, Fang Liu, Pei-Lei Zhang, Xiao-Cong Li, Jun-Gong Zhao, Hai-Tao Lu

**Affiliations:** 1 Department of Diagnostic and Interventional Radiology, Shanghai Jiao Tong University Affiliated Sixth People’s Hospital, Shanghai, China; 2 Department of Endocrinology, Shanghai Jiao Tong University Affiliated Sixth People’s Hospital, Shanghai, China; University of Bologna, ITALY

## Abstract

**Objectives:**

To evaluate the efficacy of percutaneous aspiration thrombectomy (PAT) for infrainguinal arterial thromboembolism in patients undergoing endovascular recanalization (EVR) and to investigate the predictors for thromboembolic complications.

**Materials and Methods:**

In total, 23 patients (23 limbs) who underwent PAT for thromboembolism (PAT group, PG) during EVR and 237 patients (302 limbs) who underwent successful EVR without thromboembolic complications (control group, CG) were enrolled. Immediate post-operation and follow-up outcomes were compared between the two groups. Multivariate analysis was performed to identify the predictors of thromboembolic complications. Technical success of PAT was defined as achievement of <30% residual stenosis and restoration of mTIMI grade 3.

**Results:**

The technical success rate was 95.7% in PG. After intervention, the ankle–brachial index (ABI), restoration of blood flow and improvement in dorsal/plantar arterial pulse score showed no significant differences between PG and CG. During follow-up in PG, a sustained ABI improvement was observed in 63.6% (70.9% in CG), an improvement in walking distance in 68.8% (79.9% in CG,), ulcer healing in 75.0% (71.7% in CG) and restenosis/occlusion in 31.8% (25.2% in CG). The limb salvage rate was 100% in PG (96.0% in CG), and pain relief was observed in 66.7% patients with critical limb ischaemia (81.6% in CG). Superficial femoral artery involvement [0.233; 95% confidence interval (CI), 0.108–0.461; P < 0.001], de-novo lesion occlusion (683.8; 95% CI, 36.5–12804.6; P < 0.001) and intraluminal angioplasty (118.4; 95% CI, 8.0–1758.0; P = 0.001) was associated with high incidence of thromboembolism.

**Conclusion:**

PAT is a safe and effective treatment for thromboembolism during infrainguinal arterial EVR. SFA involvement, de-novo lesion occlusion and intraluminal angioplasty may be predictors of thromboembolic complications.

## Introduction

Arterial thromboembolism is a major complication during peripheral endovascular recanalization (EVR) that seriously compromises the procedure effects, and it can be life-threatening in some cases. The reported incidence is up to 98%[1]; however, the reported incidence of thromboembolic events that can be detected on angiography and cause clinical symptoms ranges from 1.6% to 24%[1, 2]. Although surgical embolectomy is the classic and standard treatment for the management of thromboembolic complications in the lower extremity, endovascular techniques, including catheter-directed thrombolysis (CDT), percutaneous aspiration thrombectomy (PAT) and mechanical thrombectomy using dedicated peripheral arterial percutaneous thrombectomy devices, are increasingly being used for the removal of arterial emboli and restoration of blood flow[3–5]. Fogarty[6] introduced the concept of emboli removal using a catheter as early as half a century ago, CDT is often considered the first management option, while PAT is occasionally used as a supplement to CDT. However, considering that CDT is often ineffective in emboli removal because it is usually organized plaque material that embolizes, and PAT holds promise as an effective management strategy for infrainguinal arterial thromboembolism.

RETRACTED

Few studies have reported the effectiveness of PAT for acute arterial thromboembolism during lower extremity EVR [4, 7]; besides, no study has compared the clinical outcomes of patients who undergo PAT for thromboembolism during EVR and those who undergo EVR without thromboembolic complications. Furthermore, no study has analysed the lesion characteristics of patients with thromboembolic complications and the associated predictors in patients who undergo peripheral endovascular procedures. Therefore, the purpose of this study was to evaluate the effectiveness of PAT for infrainguinal arterial thromboembolism that occurred in patients undergoing EVR by comparing the lesion characteristics and clinical outcomes of these patients with those of patients without thromboembolic complications. The predictors of such thromboembolic complications were also determined.

## Materials and Methods

### Patient information

This study was conducted in accordance with the recommendations of the Declaration of Helsinki and was approved by the ethics committees of Shanghai Jiao Tong University Affiliated Sixth People’s Hospital. All patients provided written informed consent. Between January 2012 and March 2014, a total of 276 consecutive patients with lower extremity (351 limbs) arterial stenoses who underwent EVR were retrospectively analysed at our centre. 237 patients (302 limbs) successfully underwent EVR without thromboembolic complications (control group, CG). Arterial thromboembolism occurred in 23 patients (23 limbs; 6.6%), 22 (95.7%) of whom were successfully managed by PAT (PAT group, PG). Demographic, physical and clinical assessments; radiological findings, recanalization techniques and outcomes were assessed and compared between the two groups. The general condition and clinical data for the patients is outlined in Table 1.

RETRACTED

**Table 1:** Demographic characteristics, risk factors and clinical features of patients in the percutaneous aspiration thrombectomy (PAT) group (PG) and control group (CG).

Variables	PG (n = 23 limbs in 23 patients)	CG (n = 302 limbs in 237 patients)	P-value
**Age, years, mean**	68.7 ± 10.9	69.8 ± 7.7	0.531
**Gender, M (%)**	14 (60.9)	131 (55.3)	0.606
**Diabetes mellitus duration (yrs)**	10.4 ± 7.2 (n = 20, 87.0%)	13.8 ± 8.5 (n = 201, 84.8%)	0.086
**Risk factors**			
Hypertension (%)	21 (91.3)	175 (73.8)	0.109
Smoking (%)	7 (30.4)	96 (40.5)	0.346
Hyperlipidaemia (%)	2 (8.7)	17 (7.2)	1.000
Coronary artery disease (%)	7 (30.4)	46 (19.4)	0.210
Renal insufficiency (%)	4 (17.4)	23 (9.7)	0.426
**Presentation, n**			0.308
Severe claudication	16(69.6)	139(58.6)	
CLI	7(43.8)	98(41.4)	
**Duration of symptoms (months)**	1.5 ± 0.9	10.8 ± 17.3	<0.001^*^

Continuous data are presented as means ± standard deviations and categorical data as number (%).

* represents a significant difference

CLI: critical limb ischaemia

### EVR protocol

All EVR procedures in this study were performed by two experienced interventional cardiologists using a digital angiography unit (Artis Zee, Siemens, Germany) within 15 days after computed tomography angiography (CTA) or magnetic resonance angiography (MRA). The procedure was performed under local anaesthesia, and the target vessels were approached via ipsilateral, contralateral or brachial access. EVR was performed using intraluminal and/or subintimal recanalization with multiple wiring techniques in all patients, who received an average 4000-unit intravenous bolus of heparin before balloon dilatation. An additional 1000 units were administered every hour to maintain heparinization. Self-expandable stents (MARIS, Invatec S.p.A, Italy; Complete SE, Medtronic, Inc., Galway, Ireland) were placed in patients with flow-limiting dissections or residual stenosis (>30%) above the knee. DSA was performed to display vascular patency in the treated lower extremity and confirm the occurrence of thromboembolic complications.

### PAT protocol

If angiography indicated thrombosis or embolization in the treated or distal runoff after recanalization and impaired blood flow restoration, then PAT was attempted. Under roadmap guidance, a 0.035- (Terumo, Tokyo, Japan) or 0.018-inch hydrophilic guide wire (V18, Boston Scientific, Boston, MA, USA; or Hi-torque SteelCore 18, Abbott, USA) was cautiously advanced to bypass the thrombus or thromboembolus. According to the diameter of the thromboembolic segment vessel, 5F to 6F guiding catheters (ENVOY MPD, Cordis, FL, USA) were used for PAT. The guiding catheter was introduced and passed though the thromboembolic segment under support from a guidewire, and a 20- or 50-mL syringe was connected to the guiding catheter following guidewire removal. Under suction provided by a syringe, we gently and slowly withdrew the guiding catheter. Resistance by the catheter during withdrawal or sudden slowing of the blood return often indicated that the thrombus was tacked, and the catheter was completely withdrawn to check if the thrombus was sucked into the syringe or within the guiding catheter. We often directly squirted the contents in the syringe on a gauze to check for a thromboembolus. Contrast medium was injected to confirm whether the target vessel was patent and whether multiple aspirations were necessary to achieve satisfactory blood flow restoration. Following PAT, a certain amount of urokinase (250,000–500,000 U) was diluted in a 50-mL saline solution and gradually infused into the treated artery to dissolve any remaining clots in all cases, even though no clots were present angiographically. The post-intervention regime included dual anti-platelet therapy with aspirin (100 mg/d) and clopidogrel (75 g/d) for at least 3 months and lifelong aspirin (100 mg/d) therapy.

RETRACTED

### Angiography findings

The lesion characteristics evaluated in this study included lesion length and location, stenosis grade, lesion type and applied procedure techniques. On the basis of DSA images, the lesion location was classified as the superficial femoral artery (SFA), popliteal artery (PA) and infrapopliteal artery, while the stenosis grade was defined as 50%-90% stenosis, >90% stenosis and occlusion.

### Outcome evaluation and definitions

The modified thrombolysis in myocardial infarction (mTIMI) flow grade was used to assess blood flow through the thromboembolic artery immediately after PAT as follows[8]: grade 0, (no perfusion), absence of any anterograde flow beyond the occlusion; grade 1 (penetration without perfusion), faint anterograde flow beyond the occlusion with incomplete filling of the distal foot bed; grade 2 (partial reperfusion), delayed or sluggish anterograde flow with complete filling of the distal territory and grade 3 (complete perfusion), normal flow that filled the distal foot bed completely. The pulse volume score was graded on a scale from 0 to 3 as follows: 0, no palpable pulse; 1, low-grade pulse; 2, middle-grade pulse and 3, normal pulse. A 10-cm visual analogue scale (VAS) was used to assess pain levels in patients with critical leg ischaemia (CLI) before and after the procedure. An ankle–brachial index (ABI) of >0.15 and an mTIMI flow grade of >1 were defined as improvements, while a >2-cm decrease in pain level indicated pain relief. Technical success was defined as the achievement of <30% residual stenosis within the treated segment and restoration of mTIMI grade 3 flow.

RETRACTED

### Follow-up protocol

Primary patency at 12 months was defined as no re-stenosis (>50%) on Duplex ultrasound or CTA/MRA[8]. In patients with recurrent ischaemic symptoms, DSA was performed and re-intervention was attempted if necessary. An improvement in clinical symptoms (walking distance, pain relief and ulcer healing), ABI and the limb salvage rate were assessed at each follow-up visit. A decrease in ulcer size of greater than 50% was considered an improvement. Any above-ankle amputation was considered as limb salvage failure.

### Statistical analysis

Continuous variables are expressed as means ± standard deviations (SDs), while categorical variables are expressed as numbers or percentages. The grouped t-test was used to compare ABI, mTIMI flow grade and pulse volume scores between CG and PG. Lesion characteristics were compared using the chi-square test. Variables that showed a significant association with arterial thromboembolism in univariate analysis (P < 0.05) were included in multivariate logistic regression analysis. Statistical analysis was performed using the SPSS statistical software package version 20.0 (IBM, Armonk, NY). A P-value of 0.05 was considered the threshold for statistical significance.

## Results

The overall technical success rate for EVR was 92.3% (324/351 limbs). Infrainguinal arterial thromboembolism occurred in 6.6% (23/351) limbs, 95.7% (22/23) of whom were successfully managed using PAT (Figs 1 and 2). Eleven thromboembolic events (47.8%) occurred in SFA, one (4.3%) in PA and 11 (47.8%) in the infrapopliteal artery. Twenty thromboembolic events were detected after balloon dilatation, while the remaining two were detected after stent placement. After PAT, >90% patency and an mTIMI grade 3 flow were achieved in 19 thromboembolic vessels (82.6%), while 50%–90% patency was achieved in three vessels (13.0%). PAT failed to aspirate the embolus in one patient because it occurred in the dorsalis pedis artery after balloon dilatation during EVR for long-segment chronic total occlusion (CTO) in SFA. Fortunately, the posterior tibial and peroneal arteries were patent in this patient; therefore, no further treatment was attempted and no ischaemic symptoms were observed during follow-up.

RETRACTED

**Fig 1:** Thromboembolism in the right tibial–peroneal artery during endovascular recanalization (EVR) in a 78-year-old man with severe claudication since 4 months and an 11-year history of diabetes. Contrast-enhanced magnetic resonance angiography (CE-MRA) and digital subtraction angiography (DSA) images show occlusion in the right superficial femoral artery (SFA) and severe stenosis in the distal popliteal artery (PA) (A, B) (arrows). After balloon dilatation and stent placement in SFA, patency is achieved (C, D) (arrows). Thromboembolic complications are detected in the tibial–peroneal artery after balloon dilatation in distal PA (E, F and G) (arrows); therefore, percutaneous aspiration thrombectomy (PAT) is performed using a 5-French aspiration catheter. The embolus is suctioned out (H). DSA demonstrates a patent artery artery (I). Lower limb computed tomography angiography (CTA) images obtained 12 months after recanalization show patency of the right SFA and infrapopliteal arteries (J).

**Fig 2:** Thromboembolism in the left superficial femoral artery (SFA) in a 78-year-old man with severe claudication since 3 weeks. Long-segment occlusion is detected in the left SFA using contrast-enhanced magnetic resonance angiography (CE-MRA) and digital subtraction angiography (DSA) (A, B) (arrows), and severe thromboembolism after stent placement is observed in SFA (C) (arrows). Percutaneous aspiration thrombectomy (PAT) is performed and embolic material is suctioned out (D). Final angiograms show good SFA patency (E).

The baseline demographics, risk factors, clinical presentation, lesion characteristics and clinical outcomes for PG and CG are shown in Tables 1 and 2. There was no significant difference in baseline demographics, risk factors and clinical presentation between the two groups. However, compared with those in CG, the duration of symptoms in PG was shorter (1.5 ± 0.9 vs 10.8 ± 17.3 months in CG, P < 0.001), the lesions were longer (16.7 ± 8.7 cm vs 12.6 ± 6.8cm in CG, P = 0.007), the proportion of patients with SFA involvement was higher (78.3% vs 44.0% in CG, P = 0.004), the proportion of patients with complete occlusion of the de-novo lesion was higher (95.7% vs 30.5% in CG, P < 0.001) and the rate of intraluminal angioplasty was higher (95.6% vs 65.6% in CG, P = 0.006). Multivariate logistic regression analysis revealed SFA involvement [odds ratio (OR), 0.233; 95% confidence interval (CI), 0.108–0.461; P < 0.001), occlusion of the de-novo lesion (OR, 683.8; 95% CI, 36.5–12804.6; P < 0.001) and intraluminal angioplasty (OR, 118.4; 95% CI, 8.0–1758.0; P = 0.001) to be significantly associated with a high incidence of thromboembolic complications (Table 3).

RETRACTED

**Table 2:** Lesion characteristics and clinical outcomes of patients in the percutaneous aspiration thrombectomy (PAT) group (PG) and control group (CG).

Variables	PG (n = 23 limbs in 23 patients)	CG (n = 302 limbs in 237 patients)	P-value
**Lesion length(cm)**	16.7 ± 8.7	12.6 ± 6.8	0.007^*^
**Lesion location**			0.040^*^
SFA	9(39.1)	77(25.5)	
PA	3(13.0)	12(4.0)	
Infrapopliteal	3(13.0)	111(36.8)	
SFA + PA	5(21.7)	42(13.9)	
SFA + infrapopliteal	1(4.3)	14(4.6)	
PA + infrapopliteal	2(8.7)	46(15.2)	
**Stenosis grades**			0.047^*^
50%–90% stenosis	1(4.3)	74(24.5)	
>90% stenosis	11(47.8)	129(42.7)	
Occlusion	11(47.8)	99(32.8)	
**Lesion type**			0.179
De novo	16(69.6)	245(81.1)	
Recurrent	7(30.4)	57(18.9)	
**Technique**			0.025^*^
Intraluminal angioplasty	20(87.0)	185(61.3)	
Subintimal angioplasty	3(13.0)	117(38.7)	
**Embolic location**			-
SFA	11(47.8)	-	
PA	1(4.3)	-	
Infrapopliteal	11(47.8)	-	
**Embolism after balloon/stent**			-
Balloon	20(87.0)	-	
Stent	3(13.0)	-	
**Patency of target vessel after PAT**			
50%–90%	2(8.7)	-	
>90% patency	20(87.0)	-	
**Immediate clinical outcome**			
ABI improvement rate (%)	86.4 (19/22)	92.4 (279/302)	0.550
mTIMI improvement rate (%)	90.9 (20/22)	95.7 (289/302)	0.613
Arterial pulse score improvement rate (%)	86.4 (19/22)	96.4 (291/302)	0.092
**Follow-up, months, n (range)**	12 (8–18)	13 (6–22)	
ABI improvement rate (%)	63.6 (14/22)	70.9 (214/302)	0.474
Walking distance improvement rate (>2000m) in patients with claudication (%)	68.8 (11/16)	79.9 (111/139)	0.304
Pain relief rate in patients with CLI (%)	66.7 (4/6)	81.6 (80/98)	0.712
Ulcer healing rate in CLI (%)	75.0 (3/4)	71.7 (43/60)	0.969
Restenosis/occlusion rate (%)	31.8 (7/22)	25.2 (76/302)	0.490
Limb salvage rate (%)	100.0 (22/22)	96.0 (290/302)	1.000

Continuous data are presented as means ± standard deviations and categorical data as number (%).

* represents a significant difference

SFA: superficial femoral artery, PA: popliteal artery, CLI: critical limb ischaemia, ABI: ankle–brachial index, mTIMI: Modified thrombolysis in myocardial infarction

Walking distance improvement rate (>2000m) in patients with claudication (%)

**Table 3:** Multivariate logistic regression analysis for predictors for thromboembolic complications.

Variable	OR	95% CI	P value
**Duration of symptom**	0.635	0.388–1.039	0.071
**Lesion length**	1.061	0.985–1.114	0.117
**SFA involvement**	0.233	0.108–0.461	<0.001^*^
**Occlusion of de-novo lesion**	683.8	36.5–12804.6	<0.001^*^
**Intraluminal angioplasty**	118.4	8.0–1758.0	0.001^*^

OR: odds ratio; CI: confidence interval; SFA: superficial femoral artery

According to thrombus classification by Sianos et al [9], we divided 23 patients with thromboembolic complications into large thrombus burden group (15 limbs in 15 patients, LTBG) and small thrombus burden group (8 limbs in 8 patients, STBG) based on the angiographic images. Lesion characteristics and clinical outcomes of patients in the LTBG and STBG were showed in S1 Table. There was no significant difference in duration of symptom, lesion length, stenosis grade, technique and embolic location and immediate clinical outcome between LTBG and STBG. However, compared with those in STBG, the proportion of patients with SFA involvement was higher (60.0% vs 0% in CG, P = 0.002) in LTBG. Multivariate logistic regression analysis for predictors for large thrombus burden was showed in S2 Table. There was significant difference in SFA involvement between LTBG and STBG [OR = 3.051; 95% confidence interval (CI), 1.269–7.335; P = 0.013].

RETRACTED

Good blood flow restoration (mTIMI grade 3) was achieved in all patients after successful recanalization based on immediate angiography, including the 302 limbs that underwent conventional EVR and the 22 limbs that developed thromboembolic complications and were successfully managed using PAT. No significant difference was found between PG and CG in the ABI (86.4% vs 92.4%, P > 0.05), mTIMI grade (90.9% vs 95.7%, P > 0.05) and arterial pulse score improvement rates (86.4% vs 96.4%, P > 0.05). The mean follow-up duration was 12 (range, 8–18) months in PG and 12 (6–22) months in CG, and complete follow-up data were obtained from all successfully treated patients. A sustained ABI improvement was observed in 63.6% (14/22) limbs in PG and 70.9% (214/302) limbs in CG (P > 0.05). Among the patients with claudication, the walking distance increased to >2000 m in 68.8% patients in PG and 79.9% patients in CG (P > 0.05). Among the patients with CLI, pain relief was achieved in 66.7% (4/6) limbs in PG and 81.6% (8/98) limbs in CG (P > 0.05) and ulcer healing within 3 months in 75.0% (3/4) limbs in PG and 71.7% (43/60) limbs in CG (P > 0.05). Re-stenosis/occlusion was showed in 31.8% (7/22) limbs in PG and 25.2% (76/302) limbs in CG (P > 0.05). Re-intervention with balloon dilatation or stent placement was performed for six limbs in PG and 57 limbs in CG (P > 0.05) because of symptom recurrence during follow-up. The remaining recurrences were not treated because the patients did not complain of ischaemic symptoms. The limb salvage rate was 100.0% (22/22) in PG and 96.0% (290/302) in CG (P > 0.05).

## Discussion

The main findings of this study are as follows. First, PAT is a safe and effective treatment for infrainguinal arterial thromboembolism in patients undergoing EVR, and it also enables these patients to achieve clinical outcomes similar to those of patients without thromboembolic complications. Second, SFA involvement, complete occlusion of the de-novo lesion and intraluminal angioplasty may be associated with a high incidence of arterial thromboembolism during EVR.

RETRACTED

Acute arterial thromboembolism during EVR can lead to a sudden decrease in tissue perfusion and threaten the viability of the treated limb, and it is a rare but severe complication requiring immediate management. Various treatment modalities are available, including surgical revascularization, local fibrinolytic therapy, mechanical thrombectomy techniques and PAT. In terms of invasiveness, amputation rate, haemorrhagic complications and cost, PAT is a safe, rapid and effective technique for thrombus removal in patients with thromboembolic complications. Since Horvath et al.[10] suggested that small emboli occurring during PTA can be aspirated using a catheter in 1978, several studies on the clinical outcomes of PAT have been reported, with a technical success rate ranging from 87.0% to 96%[1, 4, 11]. In the present study, the technical success rate for PAT was 95.7% (22/23), which was similar to previously reported rates, and a >90% patency and an mTIMI grade 3 flow were achieved in 87.0% thromboembolic vessels after PAT. We recommend the following procedures to improve the success rate. First, the guiding catheter should be advanced under the support of a leading guidewire and roadmap guidance to avoid penetration of the subintimal passage. Second, it is not necessary to fill the syringe before removal because the embolic material is either cleared or dropped distally when blood readily enters the syringe. Third, repeat aspirations should be performed for the management of residual thromboembolisms. Fourth, when the thromboembolic and de-novo stenotic segments overlap, the operator must be aware that PAT alone will not be effective in abrogating the residual stenosis; subsequent balloon dilatation or stent placement should be considered. In this study, there was overlap between the thromboembolic and de-novo stenotic segments in 11 patients, five of whom received additional stents.

Currently, the major categories of EVR crossing techniques for lower extremity arterial occlusion include intraluminal and subintimal recanalization, and few studies have compared the rate of thromboembolic complications between the two. In a study by Young-Guk et al.[12], four patients developed distal embolisms among 54 patients who underwent conventional intraluminal angioplasty, while no patient among 52 patients who underwent subintimal angioplasty. Spiliopoulos et al.[13] reported that macroscopic particulate debris was not detected in any filter in 48 patients who underwent subintimal angioplasty or femoropopliteal CTO stenting. In this study, the rate of intraluminal angioplasty was higher in PG than in CG, and multivariate logistic regression analysis revealed that intraluminal angioplasty was associated with a significantly high incidence of thromboembolism. In addition, occlusion of the de-novo lesion was a predictor of arterial thromboembolism during EVR. Karnabatidis et al.[1] reported that CTO was positively correlated with a larger amount of captured particles (P < 0.05). In addition, histopathological examination of coronary artery CTO[14] showed that the intimal plaque in short-duration CTO was highly fibrotic with calcified lesions, while that in long-duration CTO was harder with more dense calcification. In this study, the duration of symptoms was significantly shorter in PG than in CG, which indicated that short-duration lesions are susceptible to thromboembolic complications. The primary reason for this is that short-duration lesions comprise a highly fibrotic plaque and less dense calcifications, because of which the plaque is more likely to be separated from the blood vessel.

RETRACTED

Infrainguinal arterial thromboembolism in patients undergoing EVR is a well-known and feared complication with potentially devastating clinical sequelae. Although the use of the embolic protection device (EPD) during lower extremity EVR remains controversial because of its unclear effects on the prevention of thromboembolic events, high cost, potential damage to vessels and entrapment of the filter basket, it is widely accepted in cranial and carotid interventional procedures[15–17]. In a study by Mendes et al.[16], embolic events occurred in 35 of 836 interventions (4%), including two (2%) performed with EPD and 33 (4%) performed without EPD (P > 0.05). For the safe delivery and placement of EPD, a healthy segment of vessel distal to the de-novo lesion is necessary, which may not be available in patients with peripheral arterial occlusive disease, particularly those with diabetes[18]. Moreover, when EPD is used, trauma to the vessel where the device is delivered can result in dissection, spasm or thrombosis, and operators must be aware of these potential risks and continuously visualize EPD using angiography[19]. Consequently, the use of EPD is restricted at our centre, and further research is required to define the precise role of EPD in peripheral EVR and identify patients who can benefit from the use of this device. To decrease incidence of thromboembolism, we prefer to perform PAT before balloon dilation to suction out possibly existed thromboembolic material if intraluminal technique is used, especially when the guidewire can pass de-novo occlusion lesion smoothly with almost no resistance in patients with shorter-duration lesion. Because there are limited cases in our center, the efficacy and necessity of pre-PAT has to be studied further.

RETRACTED

Our study also had limitations. On the one hand, it is unclear whether there is separated and microscopic embolus particulate caused by PAT which cannot be detected by angiography, and to avert the potential distal embolism, regularly a certain amount of urokinase saline solution is infused into the treated artery in this study. On the other hand, PAT is restricted when thromboembolism occurs in infrapopliteal and below-the-ankle artery due to the narrow vessel diameter and there is no suitable guiding catheter to manage this situation.

## Conclusions

PAT is an effective treatment for thromboembolism that occurs during infrainguinal arterial EVR. SFA involvement, complete de-novo lesion occlusion and intraluminal angioplasty may be predictors of thromboembolic complications.

## Supporting Information

S1 Table Lesion characteristics and clinical outcomes of patients in the large thrombus burden group (LTBG) and small thrombus burden group (STBG). (DOCX)

S2 Table Multivariate logistic regression analysis for predictors for large thrombus burden. (DOCX)
